# Study on the Effects of Optimized Emergency Nursing Combined with Mild Hypothermia Nursing on Neurological Prognosis, Hemodynamics, and Cytokines in Patients with Cardiac Arrest

This article has been retracted.

**DOI:** 10.1155/2022/1787312

**Published:** 2022-05-26

**Authors:** Xiaoxia Wang, Chengxia Wu

**Affiliations:** ^1^The First Affiliated Hospital, Department of Pediatrics Emergency Medicine, Hengyang Medical School, University of South China, Hengyang, Hunan 421001, China; ^2^The First Affiliated Hospital, Department of Emergency Medicine, Hengyang Medical School, University of South China, Hengyang, Hunan 421001, China

## Abstract

**Purpose:**

To study the effects of optimized emergency nursing combined with mild hypothermia nursing on neurological prognosis, hemodynamics, and cytokines in patients with cardiac arrest (CA).

**Methods:**

The medical records of 147 patients who were successfully rescued by cardiopulmonary resuscitation (CPR) after CA in our hospital were retrospectively analyzed. The 56 patients admitted in 2020 who received optimized emergency nursing were recorded as the control group; and the 91 patients admitted in 2021 who received optimized emergency nursing combined with mild hypothermia nursing were recorded as the study group. The brain function of the two groups at 72 h after return of spontaneous circulation (ROSC) was analyzed: cerebral performance category (CPC) assessment method. The neurological function of the two groups before nursing and 7, 30, and 90 d after nursing was analyzed: National Institutes of Health Stroke Scale (NISHH) score. The vital signs of the two groups after 24 h of nursing were analyzed: heart rate, spontaneous breathing rate, and blood oxygen saturation. The hemodynamic indexes of the two groups at 24 hours after nursing were analyzed: mean arterial pressure (MAP), central venous pressure (CVP), systolic blood pressure (SBP), and diastolic blood pressure (DBP). The levels of cytokines of the two groups before nursing and 7 days after nursing were analyzed: tumor necrosis factor-*α* (TNF-*α*), interleukin-6 (IL-6), and interleukin-8 (IL-8). The incidence of complications and the incidence of postresuscitation syndrome (PRS) during the nursing period were compared between the two groups.

**Results:**

72 h after ROSC, the CPC results in the study group were slightly better than those in the control group, but there was no significant difference in the number of cases of CPC Grade 1, CPC Grade 2, CPC Grade 3, CPC Grade 4, and CPC Grade 5 between the two groups (*P* > 0.05). Before nursing, there was no statistical difference in the NISHH total score between the two groups (*P* > 0.05). 7, 30, and 90 d after nursing, the NISHH total score between the two groups were lower than those before nursing, and the study group's score was lower than the control group's (*P* < 0.05). 24 h after nursing, the heart rate and spontaneous breathing rate of the study group were lower than those of the control group (*P* < 0.05), and there was no significant difference in blood oxygen saturation between the two groups (*P* > 0.05). 24 h after nursing, there was no significant difference in MAP, CVP, SBP, and DBP between the two groups (*P* > 0.05). Before nursing, there was no significant difference in the levels of TNF-*α*, IL-6, and IL-8 between the two groups (*P* > 0.05). 7 d after nursing, the levels of TNF-*α*, IL-6, and IL-8 between the two groups were lower than those before nursing, and the levels of the study group were lower than those of the control group (*P* < 0.05). During the nursing period, the total complication rates of the control group and the study group were 55.36% and 34.07%, respectively, with statistical difference (*P* < 0.05). During the nursing period, the incidences of PRS in the control group and the study group were 12.50% and 3.30%, respectively, with significant difference (*P* < 0.05).

**Conclusion:**

The application of optimized emergency nursing combined with mild hypothermia nursing in CA can effectively improve the neurological prognosis and inflammatory levels of patients and reduce the incidence of body complications and PRS.

## 1. Introduction

Cardiac arrest (CA) is a common acute and critical condition in the emergency department. Ventricular fibrillation [1], cardiac tamponade [2], pulmonary embolism [3], electrolyte abnormalities [4], drug poisoning [5], and other types of causes can be triggered. At the onset of the disease, the patient's heart beat suddenly stops and the blood uptake function suddenly disappears, which can then trigger severe hypoxia and ischemia in the tissues and organs of the whole body, the release of inflammatory factors, and the production of various metabolites, resulting in multiorgan disorders or disorders in the organism, called postcardiac arrest syndrome (PCAS) [6].

If out-of-hospital treatment is not timely, the patient can enter the death phase within minutes, and occasionally the patient can be reversed with resuscitation. With the popularization and promotion of cardiopulmonary resuscitation (CPR) technology and the continuous advancement and improvement of advanced life support, the success rate of CPR in CA patients has increased significantly, but the prognosis is still poor. Globally, CA survival rates average less than 10% and rarely reach 30% [7]. However, domestic statistics show that only 5–6% of CA patients survive after timely CPR, about 30% of CA patients have permanent brain damage after return of spontaneous circulation (ROSC), and only 1.4% had complete recovery of brain function [8]. There is growing evidence that aggressive and effective intervention after ROSC can significantly improve the survival and neurological prognosis of patients with PCAS. A study by Chan et al. [9] showed that mild hypothermia therapy (32–34 °C) for in-hospital CA patients after CPR was associated with good neurological survival [9]. In recent years, mild hypothermia therapy has gradually become the most important part of further cerebral resuscitation after ROSC in CA patients and has achieved certain results, but there are few clinical studies that combine it with optimized emergency nursing care in CA patients. In this study, the implementation value of the combined application of the two was discussed. By retrospectively analyzing the medical records of 147 patients admitted to our hospital who were successfully resuscitated by extracorporeal CPR after CA, we investigated the effects of optimized emergency nursing combined with mild hypothermia nursing on neurological prognosis, hemodynamics, and cytokines of patients.

## 2. Materials and Methods

### 2.1. Research Object

The medical records of 147 patients who were successfully rescued by CPR after CA in our hospital were retrospectively analyzed. Inclusion criteria: aged 10–60 years (9 cases of children aged 10–14 years were from the ICU ward in the hospital); in line with the American Heart Association [10] diagnosis of CA; those who were successfully rescued by extracorporeal CPR and met the 90-day follow-up period after discharge; no pulmonary infection; complete case data; and signed informed consent. Exclusion criteria: out-of-hospital CA children; patients who failed CPR rescue; patients with other malignant lesions; patients with severe organic lesions of the heart and kidneys; patients with neurological diseases or a history of mental illness; lactating or pregnant women; and clinical data loser. The 56 patients admitted in 2020 who received optimized emergency nursing were recorded as the control group; and the 91 patients admitted in 2021 who received optimized emergency nursing combined with mild hypothermia nursing were recorded as the study group. Baseline information such as age, weight, gender, triggers, and comorbidities in the control and study groups were statistically analyzed, and there was no statistical significance (*P* > 0.05) (Table 1).

### 2.2. Methods

The control group received optimized emergency nursing. The nursing process and specific work content were jointly formulated by members of our hospital's optimized emergency nursing team (composed of emergency medicine, neurology, imaging, laboratory physicians, and emergency nurses).

It is divided into ① prehospital first aid: immediate on-site assessment and measurement of vital signs upon arrival of 120 personnel, immediate extracorporeal CPR for those with cardiac arrest, i.e., extra-chest cardiac compressions, airway opening, tracheal intubation, simple ventilator-assisted ventilation, opening of intravenous access, defibrillation, etc., were given, and resuscitation drugs such as epinephrine and dopamine were given; during the transfer process, the patient's baseline information and condition were collected, and the patient's information was sent to the hospital system using the WeChat platform; ② in-hospital first aid: immediately starting the green channel after admission and sending the patient to the resuscitation room and handing over to the emergency medical care. Members of the optimized emergency nursing team immediately assessed the condition and provided emergency management and advanced life support, while explaining and communicating with the family; ③ postresuscitation nursing: after CPR, the patient was routinely given an ice cap to cool the head and maintain the brain temperature at 33∼35 °C. After 24 h, the temperature was slowly rewarmed, and when the temperature returned to normal, treatments such as reducing intracranial pressure, nutrition of brain cells, correction of water-electrolyte balance, anti-infection, and ventilator-assisted breathing were given. Vital signs were closely monitored with cardiac monitoring during this period. Criteria for CPR success: after stopping compressions, the carotid artery was still pulsating, the face and lips turned from cyanosis to ruddy, spontaneous breathing appeared, and the pupils changed from large to small and had light reflexes.

The study group received optimized emergency nursing combined with mild hypothermia nursing: prehospital first aid and in-hospital first aid nursing were the same as that of the control group. Immediately after CPR, the patient was given a cooling ice blanket and a cooling ice cap to cool the whole body. Simultaneously given with a subcold instrument (HGT-200IV; Zhuhai Hejia Medical Equipment Company), 500 ml of 95% ethanol and distilled water were added, and the water level was subject to the water level required by the display. The temperature was adjusted according to the changes in the patient's condition, such as pupils, heart rhythm, and mental status, and after the body temperature was reduced to 32∼34 °C and maintained for 24 h, the mild hypothermia nursing was discontinued. The temperature was then gradually increased to 37∼37.5 °C at a rate of 0.25∼0.5 °C/h and maintained until 72 h after the patient's ROSC. The nursing after normalization of temperature was the same as that of the control group.

### 2.3. Observation Index

#### 2.3.1. Brain Function

72 h after ROSC, the cerebral performance category (CPC) assessment method [11] was used to assess the early neurological prognosis between the two groups. There were CPC Grade 1 (good brain function), CPC Grade 2 (moderate brain disability), CPC Grade 3 (severe brain disability), CPC Grade 4 (coma/vegetative state), and CPC Grade 5 (brain death).

#### 2.3.2. Neurological Function

The National Institutes of Health Stroke Scale (NISHH) [12] scores were mainly recorded before and 7, 30, and 90 d after nursing in both the groups. It consisted of 11 dimensions: visual field (0∼3 scores), gaze (0∼2 scores), sensation (0∼2 scores), speech (0∼3 scores), facial palsy (0∼3 scores), dysarthria (0∼2 scores), limb ataxia (0∼2 scores), upper limb movement (0∼8 scores), lower limb movement (0∼8 scores), level of consciousness (0∼7 scores), and neglect (0∼2 scores). The total score was 0∼42, and the higher the score the more severe the symptoms.

#### 2.3.3. Vital Signs

Heart rate, spontaneous breathing rate, and blood oxygen saturation were analyzed in both the groups for 24 h after nursing. The testing instrument was a PICCO monitor (Beijing Shimao Medical Equipment Trading Co., Ltd.).

#### 2.3.4. Hemodynamic Indexes

Mean arterial pressure (MAP), central venous pressure (CVP), systolic blood pressure (SBP), and diastolic blood pressure (DBP) were analyzed in both the groups for 24 h after nursing.

#### 2.3.5. Cytokines

Tumor necrosis factor-*α* (TNF-*α*), interleukin-6 (IL-6), and interleukin-8 (IL-8) levels were analyzed before and 7 d after nursing in both the groups. The assay methods were all enzyme-linked immunosorbent assay, and the kits were from Shanghai Sango Biotechnology Co.

The incidences of complications and PRS during nursing in both the groups were counted.

#### 2.3.6. Statistical Methods

SPSS 22.0 was applied to analyze the statistical data, and GraphPad Prism 8.0.2.263 was applied to plot the graphs. The measurement data were expressed as ($\bar{x}$ ± *s*) with *t*-tests. Count data were expressed as (%) with *χ*^2^ tests. *P* < 0.05 was considered statistically significant.

## 3. Results

### 3.1. Comparison of CPC at 72 h after ROSC between the Two Groups

72 h after ROSC, the CPC results in the study group were slightly better than those in the control group, but there was no significant difference in the number of cases of CPC Grade 1, CPC Grade 2, CPC Grade 3, CPC Grade 4, and CPC Grade 5 between the two groups (*P* > 0.05) (Figure 1).

### 3.2. Comparison of NISHH Total Score before and after Nursing between the Two Groups

Before nursing, there was no statistical difference in the NISHH total score between the two groups (*P* > 0.05). 7, 30, and 90 d after nursing, the NISHH total scores between the two groups were lower than those before nursing, and the study group's score was lower than the control group's (*P* < 0.05) (Figure 2).

### 3.3. Comparison of Vital Signs between the Two Groups

24 h after nursing, the heart rate and spontaneous breathing rate of the study group were lower than those of the control group (*P* < 0.05), and there was no significant difference in blood oxygen saturation between the two groups (*P* > 0.05) (Figure 3).

### 3.4. Comparison of Hemodynamic Indexes between the Two Groups

24 h after nursing, there was no significant difference in MAP, CVP, SBP, and DBP between the two groups (*P* > 0.05) (Figure 4).

### 3.5. Comparison of Cytokines between the Two Groups

Before nursing, there was no significant difference in the levels of TNF-*α*, IL-6, and IL-8 between the two groups (*P* > 0.05). 7 d after nursing, the levels of TNF-*α*, IL-6, and IL-8 between the two groups were lower than those before nursing, and the levels of the study group were lower than those of the control group (*P* < 0.05) (Figure 5).

### 3.6. Comparison of Incidence of Complications between the Two Groups

During the nursing period, the total complication rates of the control group and the study group were 55.36% (31/56) and 34.07% (31/91), respectively, with statistical difference (*P* < 0.05) (Table 2 and Figure 6).

### 3.7. Comparison of Incidence of PRS between the Two Groups

During the nursing period, the incidences of PRS in the control group and the study group were 12.50% (7/56) and 3.30% (3/91), respectively, with significant difference (*P* < 0.05) (Figure 7).

## 4. Discussion

Neurological injury is a major risk factor for disability and death in CA patients in the late stages of CPR treatment. After CPR for CA, patients usually have obvious hyperthermia within 24 hours after ROSC, that is, the body temperature is higher than 37 °C. The brain is a highly temperature-dependent organ with cold tolerance, but high temperatures can create damage to patients' brain function and increase poor neurological prognosis [13]. Therefore, in order to avoid further damage to brain function and ensure the therapeutic effect after ROSC, active cooling nursing should be given clinically [14].

In this survey, 72 h after ROSC, the CPC results of the study group were slightly better than those of the control group, but there was no statistical difference in the number of CPC Grade 1, CPC Grade 2, CPC Grade 3, CPC Grade 4, and CPC Grade 5 between the two groups. At 7, 30, and 90 d after nursing, the NISHH total score in both the groups were lower than those before nursing, and the study group's score was lower than the control group's score. The comparison results suggest that optimized emergency nursing combined with mild hypothermia nursing is relatively effective in reducing brain tissue damage and improving neurological prognosis. This may be due to the fact that optimized emergency nursing in this study can contribute to shorten the prehospital delay time of patients and save the in-hospital examination and resuscitation time by transmitting the patient's medical record information to the hospital in advance and through the emergency green channel, etc. After CPR, supplemented with advanced life support such as mild hypothermia nursing, the mechanism of action may be related to the fact that hypothermia slows the rate of ATP consumption, inhibits excitatory neurotransmitter release, alters intracellular messenger activity, attenuates the associated inflammatory response and disruption of the blood-cerebrospinal fluid barrier, alters gene expression and protein synthesis, and decreases intracellular calcium ion concentration and alters glutamate receptor regulation [15, 16]. Moreover, mild hypothermia therapy can sedate the central nervous system by adding ethanol (actually a central nervous system depressant), which can put the patient in a sleep state [17]. Furthermore, in conjunction with conventional physical cooling, it can reduce the body's oxygen consumption and metabolism, improve vascular permeability, increase blood oxygen content, and promote oxygen metabolism, thereby reducing cerebral edema and pulmonary edema, so as to improve microcirculation and cardiopulmonary function [18]. The above nursing measures cooperate with each other, which can effectively maintain the patient's low-temperature state, reduce the metabolic rate of the nervous system, and reduce the damage to the nervous system caused by anaerobic metabolites during cardiac arrest, so it has a good protective effect on the prognosis of the patient's neurological function.

Mild hypothermia nursing inhibits brain cell necrosis and apoptosis and protects brain tissue by reducing brain oxygen metabolism, brain cell oxygen consumption, and oxygen radical formation through hypothermia [19]. However, it is necessary to grasp the low temperature range that is suitable for use when using it. Studies have shown that, for every 1 °C decrease in body temperature, the human metabolic rate decreases by 6 to 7% [20]. The survey showed that, 24 h after nursing, the heart rate and spontaneous breathing rate of the study group were lower than those of the control group and there was no significant difference in blood oxygen saturation, MAP, CVP, SBP, and DBP between the two groups. This shows that controlling the target temperature to a mild hypothermia state of 32–34 °C can slow down the patient's heart rate and spontaneous breathing rate to a certain extent but will not have significant adverse effects on the patient's hemodynamics and cardiopulmonary function.

Inflammatory cytokines have always been considered important risk factors for brain injury in patients with CA and have important reference significance for evaluating the degree of brain injury and neurological prognosis of patients [21]. After the occurrence of CA, the body's immune function disorder, ischemia, hypoxia, etc., can prompt the body to release a large amount of inflammatory mediators such as IL-6 and IL-8, activate the function of neutrophils, and initiate the inflammatory cascade, which in turn leads to a severe and long-lasting inflammatory response in the body [22]. TNF-*α* is a cytokine involved in the body's inflammatory response and immune response, and the higher the level, the more severe the inflammatory infiltration [23]. The survey showed that, 7 d after nursing, the levels of TNF-*α*, IL-6, and IL-8 between the two groups were lower than those before nursing, and the levels of the study group were lower than those of the control group. It shows that mild hypothermia treatment can significantly inhibit the release of inflammatory factors in the body, reduce the inflammatory cascade, and protect brain tissue.

According to previous studies, temperature too low can lead to adverse reactions such as arrhythmia, hypotension, and chills in patients [24]. The results showed that during the nursing period, the total incidence of complications in the study group was significantly lower than that in the control group, but there was no statistical difference between the items such as electrolyte disorders, irregular heartbeat, lung infection, hypotension, and hyperglycemia; the incidence of PRS in the study group was significant lower than the control group. This shows that, compared with conventional nursing methods, the mild hypothermia nursing temperature controlled at 32–34°C is suitable and will not increase the risk of adverse reactions such as electrolyte disorders, irregular heartbeat, lung infection, hypotension, and hyperglycemia in patients. On the contrary, it can reduce the incidence of adverse reactions and PRS of patients to a certain extent and improve the prognosis of patients. The reasons for this may be due to the fact that, in the process of mild hypothermia nursing, the medical and nursing staff, through the correct use of instruments, timely adjustment of the temperature of the cooling blanket and ice cap, in conjunction with cardiac monitoring during the period, closely observe the patient's pupils, body temperature, heart rhythm, and other vital signs, so that the patient's aura symptoms can be detected in a timely manner and be dealt with actively, all of which can reduce complications to a certain extent and avoid adverse outcomes.

## 5. Conclusion

The application of optimized emergency nursing combined with mild hypothermia nursing in CA can effectively improve the neurological prognosis and inflammatory levels of patients and reduce the incidence of body complications and PRS.

## Figures and Tables

**Figure 1:** Comparison of CPC at 72 h after ROSC between the two groups.

**Figure 2:** Comparison of NISHH total score before and after nursing between the two groups. Note. ^*∗*^ means *P* < 0.05 compared with the same group at the same time; and ^ means *P* < 0.05 compared with the control group at the same time.

**Figure 3:** Comparison of vital signs between the two groups. Note. ^*∗*^ indicates that there is statistical significance between the two groups. (a) Heart rate (beats/min). (b) Spontaneous breathing rate (times/min). (c) Blood oxygen saturation (%).

**Figure 4:** Comparison of hemodynamic indexes between the two groups. (a) MAP (mmHg). (b) CVP (mmH_2_O). (c) SBP (mmHg). (d) DBP (mmHg).

**Figure 5:** Comparison of cytokines between the two groups. Note. ^∗^means *P* < 0.05 compared with the same group at the same time; and ^ means *P* < 0.05 compared with the control group at the same time. (a) TNF-*α* (mg/L). (b) IL-6 (pg/mL). (c) IL-8 (pg/mL).

**Figure 6:** Comparison of the occurrence of complications between the two groups.

**Figure 7:** Comparison of the occurrence of PRS between the two groups. Note. ^*∗*^ indicates that there is statistical significance between the two groups.

**Table 1:** Comparison of baseline information between the two groups.

Group	Control group (*n* = 56)	Study group (*n* = 91)	t/*χ*^2^	*P*
Age ($\bar{x}$ ± *s*, years)	39.52 ± 10.15	39.29 ± 10.19		
Weight ($\bar{x}$ ± *s*, kg)	56.84 ± 10.45	59.52 ± 10.26	1.527	0.129

Case distribution (n, %)				
Children	3 (5.36)	6 (6.59)	0.092	0.761
Adults	53 (94.64)	85 (93.41)		

Gender (*n*, %)				
Male	35 (62.50)	54 (59.34)	0.145	0.704
Female	21 (37.50)	37 (40.66)		

Triggers (*n*, %)				
Primary heart disease	26 (46.43)	42 (46.15)	0.001	0.974
Extra-cardiac disorders	30 (53.57)	49 (53.85)		

Comorbidities (*n*, %)				
Hypertension	28 (50.00)	47 (51.65)	0.038	0.846
Diabetes	15 (26.79)	26 (28.57)	0.055	0.815
Others	17 (30.36)	26 (28.57)	0.053	0.817

**Table 2:** Comparison of incidence of complications between the two groups (*n*, %).

Group	Electrolyte disorders	Irregular heartbeat	Lung infection	Hypotension	Hyperglycemia	Others	Total
Control group (*n* = 56)	10 (17.86)	8 (14.29)	2 (3.57)	3 (5.36)	2 (3.57)	6 (10.71)	31 (55.36)
Study group (*n* = 91)	11 (12.09)	5 (5.49)	2 (2.20)	4 (4.40)	2 (2.20)	7 (7.69)	31 (34.07)
*χ* ^2^	0.942	3.324	0.247	0.071	0.247	0.393	6.444
*P*	0.332	0.068	0.619	0.790	0.619	0.531	0.011

## Data Availability

The data used or analyzed during the study are available from the corresponding authors.
